# The Predominance of a Specific Genotype of *Cryptococcus neoformans* var. *Grubii* in China and Japan

This article has been retracted.

**DOI:** 10.1155/2022/8162096

**Published:** 2022-08-05

**Authors:** Jian Zhu, Jiafei Cao, Tingying Li, Qi Liu, Yingqian Kang, Zhenghong Chen, Wieland Meyer, Yuzuru Mikami, Mei Long

**Affiliations:** ^1^Department of Gastroenterology, Guizhou Provincial Orthopedic Hospital, Guiyang, Guizhou 550014, China; ^2^Department of Gastroenterology, The Affiliated Hospital of Guizhou Medical University, Guiyang, Guizhou 550004, China; ^3^Department of Pediatrics, Guiyang Second People Hospital, Guiyang, Guizhou 550081, China; ^4^Department of Microbiology, School of Basic Medical Science, Guizhou Medical University, Key Laboratory of Medical Microbiology and Parasitology of Guizhou Province, Guiyang, Guizhou 550025, China; ^5^Molecular Mycology Research Laboratory, Centre for Infectious Diseases and Microbiology, Sydney Medical School-Westmead Hospital (Research and Education Network), Marie Bashir Institute for Infectious Diseases and Biosecurity, The University of Sydney, Westmead Institute for Medical Research, Sydney, Australia; ^6^Medical Mycology Research Center (MMRC), Chiba University, China

## Abstract

**Background:**

The extensive deployment of molecular genotyping methods is the top reliable keyword to characterize the population genetic structure of *C. neoformans* in the past decade. However, studies involving genotypic analysis of *C. neoformans* var. *grubii* from China and Japan are limited.

**Objectives:**

We address this challenge to determine the genotype distribution of *C. neoformans* var. *grubii* strains from China and Japan.

**Methods:**

Genotypic analysis of 52 *C. neoformans* var. *grubii* isolates was performed using multilocus microsatellite typing (MLMT) based on the sequence analysis of 3 functional genes. In order to place the herein-studied strains into the global picture, 22 strains randomly selected from the 52 strains studied by MLMT were also analyzed by restriction fragment length polymorphism analysis of the orotidine monophosphate pyrophosphorylase gene (*URA5*-RFLP), M13 PCR-fingerprinting, and multilocus sequence typing (MLST).

**Results:**

MLMT classified 46 (88.5%) of the 52 strains as genotype MLMT-17. The high prevalence of the MLMT-17 type was observed for environmental and clinical isolates from China and Japan. *URA5*-RFLP analysis, M13 PCR-fingerprinting, and MLST showed that most of these belong to the VNI/ST5 (M5) genotype.

**Conclusions:**

Our study suggests the predominance of a specific genotype of *C. neoformans* var. *grubii* in China and Japan.

## 1. Introduction

Members of the *Cryptococcus neoformans/C. gattii* species complex are basidiomycetous yeasts, which are the etiological agents of cryptococcosis [1]. Among such opportunistic pathogens, many microbial phenotypes have been clearly correlated with virulence, including polysaccharide capsule production, formation of melanin, and secretion of various proteins [2]. The infection proceeds by inhalation and spreads to the central nervous system causing meningitis. Cryptococcosis caused by *C. neoformans* is predominantly AIDS, while infections caused by *C. gattii* often occur in immunocompetent patients [3]. The species complex is classified into two species: *C. neoformans* (serotypes A, D, and AD) and *C. gattii* (serotypes B and C) [4]. *C. neoformans* is divided into two varieties and one hybrid, namely, *C. neoformans* var. *grubii* (serotype A), *C. neoformans* var. *neoformans* (serotype D), and a hybrid of both varieties (serotype AD). More recently, it was suggested to separate the *Cryptococcus neoformans/C. gattii* species complex into seven species [1], but for this study, the traditional classification was followed. *C. neoformans* var. *grubii* has been isolated worldwide [4–8] and causes most of the cryptococcal infections in HIV-infected patients [9]. *Cryptococcus* species typically reside in a variety of environmental niches, mainly old avian droppings (especially aged pigeon droppings) [4, 5, 10, 11], decaying wood [12–14], and soil contaminated with these droppings and/or decaying wood alone [10, 13].

Several studies have focused on the molecular determinants of the number of genetically diverse subgroups within each serotype [15–18]. Molecular methods employed to define these subgroups revealed associations between geographic origin and particular genotypes, implying an epidemiologic significance of specific genotypes. Although, in the past decade, molecular genotyping methods have been applied extensively to characterize the population genetic structure of *C. neoformans*, only a few reports have been published on genotype analyses of *C. neoformans* var. *grubii* from China and Japan [19–23]. Therefore, we were prompted to conduct a genetic characterization of *C. neoformans* var. *grubii* in China and Japan using previously established microsatellite markers [17]. Microsatellites, also known as simple sequence repeats (SSR) or short tandem repeats (STRs), are highly polymorphic and spread throughout all genomes, including humans, lower eukaryotes, and fungi [24, 25]. We have previously reported the usefulness of multilocus microsatellite typing (MLMT) using three specific microsatellite-amplifying PCR primer sets (CNG1, CNG2, and CNG3) for the characterization of the genotype structure of *C. neoformans* var. *grubii* [17, 26]. To date, 38 MLMT types have been recognized globally among *C. neoformans* var. *grubii* isolates [17].

In the current study, we applied MLMT to characterize the genotypes of 52 strains isolated in China and Japan. To place the Chinese and Japanese cryptococcal isolates in a global context and to compare the herein used MLMT typing technique with the typing techniques used elsewhere, 22 of 52 Chinese and Japanese strains were randomly selected and subjected to the restriction fragment length polymorphism analysis of the orotidine monophosphate pyrophosphorylase gene *(URA5-*RFLP), M13 PCR-fingerprinting, and multilocus sequence typing (MLST) analysis.

## 2. Methods

### 2.1. Ethics Statement

This study was approved by the institutional ethics committee (Guiyang Hospital of Guizhou Aviation Industry Group Research Ethics Committee, permission number: 2015-037).

### 2.2. PCR Amplification, DNA Sequencing, and Multilocus Microsatellite Typing (MLMT)

#### 2.2.1. Strains Used

Thirty-nine isolates of *C. neoformans* var. *grubii* from China (including 30 clinical isolates, eight environmental isolates, and one isolate from an unknown source) and 13 isolates from Japan (6 clinical isolates and seven isolates from unknown sources) were studied (Table 1). Of the strains isolated in China, seven were from Beijing, nine (including five environmental strains) from Nanjing, five from Shanghai, and 15 from Guangzhou, including three environmental strains. All of the environmental strains were isolated from pigeon droppings in China. Of the 13 isolates collected in Japan, seven were from Chiba Prefecture (central Japan), and six were from Nagasaki Prefecture (western Japan) (Table 1). Clinical samples included CSF (cerebrospinal fluid, 25 strains), BAL (bronchial lavage, three strains), TBLB (transbronchial lung biopsy, one strain), and sputum (one strain). All strains were initially identified as *C. neoformans* by standard microbiological methods and growth characteristics on Canavanine-Glycine-Bromothymol blue (CGB) agar [27]. The strains were grown on potato dextrose agar (PDA, Difco Laboratories, Detroit, MI, USA) slants and incubated at 30°C for 48–72 h before DNA extraction.

#### 2.2.2. DNA Extraction

Genomic DNA was extracted as previously described [26]. Briefly, 3–4 loops of yeast cells from PDA slants were suspended in TE buffer (10 mmol L^−1^ Tris-HCl, 1 mmol L^−1^ EDTA, and pH 8.0). Tris-HCl (pH 8.0) was added to the washed yeast cells and boiled. After treatment with chloroform-isoamyl alcohol, the aqueous phase was separated. The aqueous layer was mixed with isopropanol and 3 mL ammonium acetate. The samples were centrifuged, and the resulting nucleic acid pellets were washed, dried, and finally resuspended in TE buffer.

#### 2.2.3. PCR for Mating-Type Determination

The mating type was determined according to Halliday and Carter [28] using specific primers for the amplification of both *a* and *α* loci.

#### 2.2.4. MT Analysis

MT types were determined as previously reported [17, 26]. Namely, PCR primers, which amplify three microsatellite loci, designated CNG1, CNG2, and CNG3, were used. The microsatellite locus CNG1 has repeats of the “TA” motif, with repeat numbers ranging from 9 to 13, resulting in five microsatellite allele types. The locus CNG2 has reproductions of the “GA” motif, with repeat numbers ranging from 7 to 12, resulting in 6 microsatellite allele types. Finally, the microsatellite locus CNG3 has repeats of the “CAT” motif, with repeat numbers ranging from 5 to 12, resulting in 8 microsatellite allele types. These microsatellites were amplified using Ready-To-Go PCR beads (Amersham Pharmacia Co., Piscataway, NJ, USA), a set of primers (CNG1, CNG2, and CNG3) at a final concentration of 1 *μ*M, and 25 pg of genomic DNA, in a volume of 25 *μ*L using a GeneAmp 9600 thermocycler (Perkin-Elmer Inc., USA). The PCR conditions were as previously described [17, 26]. The amplified PCR products were purified using a PCR product pre-sequencing kit (ExoSAP-IT; USA Corp., Cleveland, OH, USA), and the DNA sequences were determined by an automatic sequencer (ABI PRISM™ 3100; PE Applied Biosystems, Tokyo, Japan). MLMT allele types were determined by calculating the number of repeats in each locus, and the MLMT type was determined by combining the repeat allele numbers of the three different motifs [26].

### 2.3. RA5-RFLP, M13 PCR-Fingerprinting, and MLST Analysis Using the ISHAM Consensus MLST Scheme for the C. neoformans/C. gattii Species Complex

#### 2.3.1. Used

To place the Chinese and Japanese strains in a global context, 22 out of the 52 strains used in MLMT analysis were randomly selected from the cultures isolated in China and Japan. In addition, the following standard strains of the eight major molecular types of the *C. neoformans/C. gattii* species complex have been included for significant molecular type identification: WM148 (VNI, serotype A, CSF, HIV-, Australia), WM626 (VNII, serotype A, CSF, HIV-, Australia), WM628 (VNIII, serotype AD, CSF, HIV+, Australia), WM629 (VNIV, serotype D, Blood, HIV+, Australia), WM179 (VGI, serotype B, CSF, HIV-, Australia), WM178 (VGII, serotype B, CSF, HIV-, Australia), WM175 (VGIII, serotype B, Eucalypt, USA), and WM779 (VGIV, serotype C, Cheetah, South Africa).

#### 2.3.2. DNA Extraction

For DNA extraction, the strains were grown on Sabouraud dextrose agar slants at 37°C for two days. Then, the cells were collected by centrifugation, and the cell pellets were frozen in liquid nitrogen. The frozen cells were ground with a miniature pestle (1.5 cm diameter). The tubes were kept in the freezer at −20°C overnight, and ground cells were mixed with lysis buffer and 2-mercaptoethanol. The samples were mixed vigorously and then incubated at 65°C for 1 h (vortexed at least once during incubation). DNA was extracted as described previously [29].

#### 2.3.3. *URA5*-RFLP *Analysis*

PCR amplification of the *URA5* gene was conducted using the forward primer URA5 (5′-ATGTCCTCCCAAGCCCTTCGACTCCG-3′), and the reverse primer SJO1 (5′-TTAAGAC CTCTGAACACCGTACTC-3′) as previously described [30]. A portion of the PCR products was then double digested with the restriction enzymes *Sau*961 and *Hha*I. The digestion products were separated on a 3% agarose gel. The major molecular types were determined by manual comparison with the RFLP patterns of standard strains of the eight major molecular types.

#### 2.3.4. M13 PCR-Fingerprinting

Strain typing was performed using PCR-fingerprinting with the core sequence of the wild-type phage M13-specific primer (5′-GAGGGTGGCGGTTCT-3′) [7] using 10 ng *μ*L^−1^ genomic DNA and Ready-To-Go PCR beads (Amersham Pharmacia Co., Piscataway, NJ, USA) in a volume of 25 *μ*L as previously illustrated [30, 31]. The main molecular types were determined by manual comparison with the PCR-fingerprinting patterns of standard strains of the eight major molecular types. Strain genotypes were identified based on their individual banding patterns.

#### 2.3.5. MLST Analysis

Strains were randomly selected for MLST analysis based on seven unlinked loci, i.e., *CAP59*, which encodes a capsular-associated protein; *GPD1*, which encodes glyceraldehyde-3-phosphate dehydrogenase; IGS1, which encodes a ribosomal RNA intergenic spacer; *LASC1*, which encodes laccase; *PLB1*, which encodes phospholipase; *SOD1*, which encodes Cu, Zn superoxide dismutase; and *URA5*, which encodes orotidine monophosphate pyrophosphorylase. Each genetic locus was amplified using the primers and amplification parameters described by the International Society for Human and Animal Mycology (ISHAM) Cryptococcal Working Group for genotyping *C. neoformans and C. gattii* and analyzed as previously reported [32, 33]. Allele and sequence types were determined against the MLST webpage of the University of Sydney (https://mlst.mycologylab.org).

## 3. Results

### 3.1. Distribution of the MLMT Types of C. neoformans var. Grubii Strains in Chinese and Japanese Cultures

Based on the repeat numbers of each microsatellite, the combined MLMT types were determined and are shown in Table 1. The 52 *C. neoformans* var. *grubii* strains were classified into 7 MLMT types (MLMT-2, MLMT-14, MLMT-16, MLMT-17, MLMT-29, MLMT-34, and MLMT-39), with the major one being MLMT-17 (88.5%, 46 out of the 52 strains). MLMT-39 was identified as a novel MLMT type with a unique SSR allele at the microsatellite region in CNG1 (DDBJ accession number AB488809). The most common repeat number of the “TA” motif of the microsatellite locus CNG1 was 12, and 46 strains belong to this repeat number group in MLMT-17. However, the number of repeats of the “GA” and “CAT” motifs of the microsatellite loci of CNG2 and CNG3 in MLMT-17 was 12 and 7, respectively, and 49 and 50 out of the 52 strains, respectively, presented these repeat numbers. The distribution of the MLMT types in Chinese and Japanese cultures is shown in Figure 1(a), in comparison with the MLMT types obtained globally (except for cultures from China, Brazil, and Japan; Figure 1(b)), and the MLMT types obtained from Brazilian cultures are shown in Figure 1(c). Among the 52 strains, 39 Chinese isolates were classified into 6 MLMT types: MLMT-14 (1 strain), MLMT-16 (1 strain), MLMT-17 (34 strains), MLMT-29 (1 strain), MLMT-34 (1 strain), and MLMT-39 (1 strain). The regional MLMT-type distribution patterns of the Chinese isolates are shown in Figure 2. Thirteen Japanese isolates were classified into 2 MLMT types, namely, MLMT-2 (1 strain) and MLMT-17 (12 strains), with the latter MLMT type being predominant amongst the Japanese isolates studied. The MLMT-17 type was highly prevalent in both countries, with prevalence ratios being in China at 87.2% and Japan at 92.3%.

### 3.2. High Prevalence of the MLMT-17 Type in China and Japan

Information on the 36 strains from patients, including 25 strains from CSF, three strains from BAL, one strain from TBLB, and one strain from sputum, is shown in Table 1. For the remaining nine strains, no patient information was available. A correlation analysis between clinical status and MLMT type revealed that the MLMT-17 type predominates the clinical samples regardless of their isolation site. Out of the eight environmental isolates, seven strains were of the MLMT-17 type (87.5%), being the major type in Chinese and Japanese pigeon droppings. The remaining strain was of the MLMT-29 type.

### 3.3. VNI/ST5(M5) Is One Specific Genotype among Chinese and Japanese C. neoformans var. Grubii Isolates

To compare the herein applied typing method to other typing methods and to place them into the global molecular epidemiology of the *C. neoformans/C. gattii* species complex, 22 randomly selected strains from the 52 *C. neoformans* var. *grubii* isolates from China and Japan were studied for MLMT typing and subjected to *URA5*-RFLP analysis, M13 PCR-fingerprinting, and MLST typing (Table 2). *URA5*-RFLP analysis showed that all 22 isolates were of molecular type VNI (Table 2). PCR-fingerprinting using the minisatellite specific primer M13 showed a significant pattern that is shared among most of the studied isolates. The pattern can be seen in all 22 VNI isolates. MLST of the 22 strains for seven loci revealed the presence of a predominant MLST type, VNI/ST5 (M5), to which 19 of the isolates (86%) belonged. The results of MLST typing compared to those of the MLMT typing are shown in Table 2, confirming the predominance of one specific genotype among Chinese and Japanese *C. neoformans* var. *grubii* isolates.

Strain IFM 47272 belongs to the MLST type ST32 (M4) (MLMT-14), and strain IFM 45722 belongs to the MLST type ST31 (M4b) (MLMT-29). One of the isolates, IFM 40045, represents a novel, previously unidentified MLST sequence type ST66 (MLMT-2). The strains IFM 45721, IFM 45726, and IFM 52370 belong to the same MLST type as ST5 (M5), but they were classified into different MLMT types, namely, MLMT-39, MLMT-34, and MLMT-16, respectively (Table 2).

## 4. Discussion

Studies have previously reported the usefulness of MLMT using the sequences of three different microsatellite regions for the genotyping of *C. neoformans* isolates [17, 26]. To date, 176 strains of *C. neoformans* var. *grubii* have been classified into 38 MLMT types [17, 26]. In the present study, newly isolated 52 strains of the *C. neoformans* var. *grubii* from China and Japan were classified into 7 MLMT types using the same MLMT method. Most of these (46 strains) were classified into one major genotype, MLMT-17 (88.6%). In both countries, the MLMT-17 type was highly prevalent. The prevalence ratios of MLMT-17 in China were 87.2% and Japan at 92.3%, suggesting that clonal reproduction among the populations of *C. neoformans* var. *grubii* in the two countries may be the main reproductive style. This was also previously observed in Taiwan, where two isolates of *C. neoformans* var. *grubii* were classified as the MLMT-17 type [26]. There was only one allele type difference between the major type (MLMT-17) and the three other types (MLMT-16, MLMT-29, and MLMT-39), indicating that these are genetically very closely related. Therefore, microevolution in *C. neoformans* var. *grubii* strains in China and Japan might be a reasonable explanation for the presence of MLMT-16, MLMT-29, and MLMT-39 [34]. These results suggest a predominance of one specific MLMT type (MLMT-17) among the Chinese and Japanese isolates.

Furthermore, strain IFM 45772 (MLMT-29) was classified as VNI according to major molecular type and pattern. It differed from MLST type ST5 (M5) and was classified as MLST type ST31 (M4b) due to sequence differences in the *GPD1*, *IGS1*, and *LAC1* loci. Further studies on the strains of the MLMT-29 type are essential, considering that the strain IFM 45772 was isolated from pigeon droppings. In contrast, the isolation sites of the three previously studied strains are unknown [26]. The remaining type MLMT-2 is different from MLMT-17 in terms of sequences of two loci, CNG1 and CNG2. We previously isolated MLMT-2 from Costa Rica [26]. In addition, we also reported about 12 strains belonging to the MLMT-2 type from pigeon droppings and clinical samples from Brazil [26]. As such, strains of the MLMT-2 genotype are also considered to be widely distributed in South and Central America as well as East Asia. Finally, the strain IFM 47272 with the genotype MLMT-14 was isolated in China. This genotype was previously isolated from Brazil (2 strains), again suggesting a wide distribution.

In addition, we found that MLMT typing and M13 PCR-fingerprinting are highly concordant. Our results agree well with a report in which most of the Chinese strains of the *C. neoformans* var. *grubii* belong to one particular group, which was based on M13 PCR-fingerprinting [21]. In addition to the application of MLMT to typing strains of the haploid major molecular types of *C. neoformans*, we also found that AD hybrid strains show different profiles of the CNG1, CNG2, and CNG3 loci, which are easily differentiated from those of the haploid *C. neoformans* var. *grubii* strains (data not shown). Therefore, it is possible to determine the AD hybrid strains from the haploid *C. neoformans* var. *grubii* strains by MLMT typing. The present results also persistently encourage the hypothesis that human cryptococcosis can be acquired from an immediate environmental reservoir, based on the isolation of the MLMT-17 type from patients and the environment, such as pigeon droppings [5, 11, 30].

Also, M13 PCR-fingerprinting illustrated that most of the studied strains (86.4%) exhibited an identical band pattern, the VNI clade, which includes the clinic and environmental isolates. MLST analysis also revealed a common sequence type (86.4%), ST5 (M5). Three out of the four environmental isolates that were recovered from pigeon excreta also belonged to the sequence type ST5 (M5). This suggests that cryptococcal infections in Chinese patients could be due to the inhalation of cryptococcal cell-contaminated droplets from pigeon excreta. However, more environmental samples should be studied to verify the source of the infection undoubtedly. MLST analysis of strain IFM 47272 revealed that this isolate belongs to the sequence type ST32 (M4). The sequence alignment of the 7 MLST loci showed an identical pattern to the international reference strain br795 isolated in Brazil, which belongs to the MLMT-14 type [17]. Therefore, further detailed environmental studies of the isolation site are warranted, as, currently, only two strains are available. MLST analysis of the isolate IFM 45722 (MLMT-29) showed that it is identical with sequence type M4b and is grouped with the international reference strain ug2471, which we assessed in our previous study [26] where we isolated three strains of this genotype in Japan. The isolate IFM 40045 (MLMT-2) did not group with any of the reference strains for the MLST locus *LAC1* and was subsequently identified as a new sequence type. However, MLMT typing confirmed the presence of this genotype in Brazil and Costa Rica [17].

Recent multi-institutional studies by Chen et al. [21], Khayhan et al. [31], and Kaocharoen et al. [6] revealed that the Asian *C. neoformans* var. *grubii* populations of Thailand, China, and Japan show limited genetic diversity and demonstrate a largely clonal mode of reproduction compared to the global MLST dataset. These reports suggest that ST5 (M5) is the major MLST genotype among *C. neoformans* var. *grubii* isolates in China and Japan, and the sequence types ST4 (M4) and ST6 (M6) are more predominant in Thailand [6, 30]. High distribution ratios of *C. neoformans* var. *grubii* strains with the MLST type ST5 (M5) in Japan were also recently reported by Umeyama et al. [35] and Mihara et al. [36]. The prevalence of the ST5 (M5) genotype of *C. neoformans* var. *grubii* in Korea was also reported by Park et al. [37] Furthermore, the Asian population of *C. neoformans* var. *grubii* has been shown to be genetically less diverse than those occurring in Africa [38, 39] and Europe [40], and one genotype is predominant in China [21, 22]. In this study, the presented analysis using MLMT confirmed the predominant distribution of a specific genotype MLMT-17/VNI/ST5 (M5) in China and Japan, reinforcing the findings of recent reports [6, 21, 22, 35, 36].

Some studies [9, 26, 41] have indicated that due to the burden of HIV infection, its associated cryptococcosis is more prevalent in other countries, especially in South Africa. And with increasing immigration, more subtypes of *C. neoformans* var. *grubii* would emerge. Although the situation in China is considered to be more complex, further analysis by MLMT typing using more extensive samples from clinical and environmental sources in China and Japan is needed to improve our understanding of the infection route of cryptococcosis in these countries.

## 5. Conclusion

In conclusion, We identified for the first time that a predominant distribution of a specific genotype of *C. neoformans* var. *grubii*, MLMT-17/VNI/ST5 (M5) in China and Japan. This genotype is also considered as the major genotype among Asian countries, but more general conclusions require more extensive investigations. Continuous monitoring of the genotype distribution of cryptococcosis is important for the investigation of HIV-associated cryptococcosis in Asian countries.

## Figures and Tables

**Figure 1:** MLMT-type distribution of *Cryptococcus neoformans* var. *grubii* isolates. (a) MLMT-type distribution of 52 Chinese and Japanese *Cryptococcus neoformans* var. *grubii* isolates. (b) MLMT-type distribution of 87 global strains of *Cryptococcus neoformans* var. *grubii* (modified data from 27), excluding Brazilian, Chinese, and Japanese isolates. (c) MLMT-type distribution among 89 Brazilian *Cryptococcus neoformans* var. *grubii* strains (modified data from Zhu et al. [17]). MLMT: multilocus microsatellite typing.

**Figure 2:** MLMT-type distribution of 39 *Cryptococcus neoformans* var. *grubii* strains isolated from Beijing, Guangzhou, Nanjing, Shanghai, and Guiyang in China. MLMT: multilocus microsatellite typing.

**Table 1:** List of *Cryptococcus neoformans* var. *grubii* strains studied, their sources, country of origin, CNG-Allele type, and multilocus microsatellite type (MLMT).

IFM strain number	Source of isolation	Country of origin	CNG1 allele type (TA repeat number)	CNG2 allele type (GA repeat number)	CNG3 allele type (CAT repeat number)	MLMT type
45835 (WM09.168)	Unknown	CH, Japan	3 (12)	5 (12)	2 (7)	17
45836	Unknown	CH, Japan	3 (12)	5 (12)	2 (7)	17
45839	Unknown	CH, Japan	3 (12)	5 (12)	2 (7)	17
45840	Unknown	CH, Japan	3 (12)	5 (12)	2 (7)	17
45841	Unknown	CH, Japan	3 (12)	5 (12)	2 (7)	17
45842 (WM09.169)	Patient	CH, Japan	3 (12)	5 (12)	2 (7)	17
45843	Unknown	CH, Japan	3 (12)	5 (12)	2 (7)	17
40045 (WM09.170)	Unknown	N, Japan	1 (9)	3 (10)	2 (7)	2
46652 (WM09.171)	Sputum	N, Japan	3 (12)	5 (12)	2 (7)	17
46654	TBLB	N, Japan	3 (12)	5 (12)	2 (7)	17
46655 (WM09.172)	CSF	N, Japan	3 (12)	5 (12)	2 (7)	17
46658	BAL	N, Japan	3 (12)	5 (12)	2 (7)	17
59	BAL	N, Japan	3 (12)	5 (12)	2 (7)	17
55983 (WM09.173)	CSF	BJ, China	3 (12)	5 (12)	2 (7)	17
55984	CSF	BJ, China	3 (12)	5 (12)	2 (7)	17
55985	CSF	BJ, China	3 (12)	5 (12)	2 (7)	17
55986 (WM09.174)	CSF	BJ, China	3 (12)	5 (12)	2 (7)	17
55987	CSF	BJ, China	3 (12)	5 (12)	2 (7)	17
56847 (WM09.176)	CSF	GZ, China	3 (12)	5 (12)	2 (7)	17
56848	CSF	GZ, China	3 (12)	5 (12)	2 (7)	17
56849	CSF	GZ, China	3 (12)	5 (12)	2 (7)	17
56850 (WM09.177)	CSF	GZ, China	3 (12)	5 (12)	2 (7)	17
56851	CSF	GZ, China	3 (12)	5 (12)	2 (7)	17
45712	CSF	NJ, China	3 (12)	5 (12)	2 (7)	17
45717 (WM09.181)	CSF	NJ, China	3 (12)	5 (12)	2 (7)	17
47272 (WM090.175)	CSF	BJ, China	2 (11)	5 (12)	6 (12)	14
47273	CSF	BJ, China	3 (12)	5 (12)	2 (7)	17
45721 (WM09.178)	Patient	SH, China	5 (14)	5 (12)	2 (7)	39
45722	Patient	SH, China	3 (12)	5 (12)	2 (7)	17
45723 (WM09.179)	Patient	SH, China	3 (12)	5 (12)	2 (7)	17
45725	Patient	SH, China	3 (12)	5 (12)	2 (7)	17
45726 (WM09.180)	Patient	SH, China	1 (9)	3 (10)	1 (5)	34
45760	Pigeon dropping	NJ, China	3 (12)	5 (12)	2 (7)	17
45764 (WM09.185)	Pigeon dropping	NJ, China	3 (12)	5 (12)	2 (7)	17
45766 (WM09.186)	Pigeon dropping	NJ, China	3 (12)	5 (12)	2 (7)	17
45768	Pigeon dropping	NJ, China	3 (12)	5 (12)	2 (7)	17
45772 (WM09.187)	Pigeon dropping	NJ, China	4 (13)	5 (12)	2 (7)	29
52696 (WM09.188)	BAL	GZ, China	3 (12)	5 (12)	2 (7)	17
52364 (WM09.189)	CSF	GZ, China	3 (12)	5 (12)	2 (7)	17
52366	CSF	GZ, China	3 (12)	5 (12)	2 (7)	17
52368	CSF	GZ, China	3 (12)	5 (12)	2 (7)	17
52370 (WM09.190)	CSF	GZ, China	3 (12)	4 (11)	2 (7)	16
52372	CSF	GZ, China	3 (12)	5 (12)	2 (7)	17
52376	CSF	GZ, China	3 (12)	5 (12)	2 (7)	17
52378	CSF	GZ, China	3 (12)	5 (12)	2 (7)	17
52379	CSF	GZ, China	3 (12)	5 (12)	2 (7)	17
52380	CSF	GZ, China	3 (12)	5 (12)	2 (7)	17
45718 (WM09.182)	CSF	NJ, China	3 (12)	5 (12)	2 (7)	17
48163	Unknown	NJ, China	3 (12)	5 (12)	2 (7)	17
57499 (WM09.191)	Pigeon dropping	GY, China	3 (12)	5 (12)	2 (7)	17
57500	Pigeon dropping	GY, China	3 (12)	5 (12)	2 (7)	17
57502	Pigeon dropping	GY, China	3 (12)	5 (12)	2 (7)	17

BAL: bronchial lavage; TBLB: transbronchial lung biopsy; CSF: cerebrospinal fluid; BJ: Beijing; CH: Chiba; GY: Guiyang; GZ: Guangzhou; N: Nagasaki; NJ: Nanjing; SH: Shanghai.

**Table 2:** ISHAM consensus scheme MLST types of selected Chinese and Japanese strains in comparison with the MLST types obtained previously, the MLMT types, and the *URA5*-RFLP patterns.

Strain no.	IFM no	*CAP59*	*GPD1*	IGS1	*LAC1*	*PLB1*	*SOD1*	*URA5*	MLST ST^#^	MLST type∗	MLMT type	Major molecular type^1^
WM09.168	45835	1	3	1	5	2	1	1	5	M5	17	VNI
WM09.169	45842	1	3	1	5	2	1	1	5	M5	17	VNI
WM09.170	40045	7	1	1	12	1	1	2	66		2	VNI
WM09.171	46652	1	3	1	5	2	1	1	5	M5	17	VNI
WM09.172	46655	1	3	1	5	2	1	1	5	M5	17	VNI
WM09.173	55983	1	3	1	5	2	1	1	5	M5	17	VNI
WM09.174	55986	1	3	1	5	2	1	1	5	M5	17	VNI
WM09.175	47272	1	1	10	3	4	1	1	32	M4	14	VNI
WM09.176	56847	1	3	1	5	2	1	1	5	M5	17	VNI
WM09.177	56850	1	3	1	5	2	1	1	5	M5	17	VNI
WM09.178	45721	1	3	1	5	2	1	1	5	M5	39	VNI
WM09.179	45723	1	3	1	5	2	1	1	5	M5	17	VNI
WM09.180	45726	1	3	1	5	2	1	1	5	M5	34	VNI
WM09.181	45717	1	3	1	5	2	1	1	5	M5	17	VNI
WM09.182	45718	1	3	1	5	2	1	1	5	M5	17	VNI
WM09.185	45764	1	3	1	5	2	1	1	5	M5	17	VNI
WM09.186	45766	1	3	1	5	2	1	1	5	M5	17	VNI
WM09.187	45772	1	1	10	3	2	1	1	31	M4b	29	VNI
WM09.188	52696	1	3	1	5	2	1	1	5	M5	17	VNI
WM09.189	52364	1	3	1	5	2	1	1	5	M5	17	VNI
WM09.190	52370	1	3	1	5	2	1	1	5	M5	17	VNI
WM09.191	57499	1	3	1	5	2	1	1	5	M5	16	VNI
c48		1	3	1	5	2	1	1	5	M5		VNI
jp1088		1	3	1	5	2	1	1	5	M5		VNI
A3 11		7	1	1	2	1	1	2	23	M3		VNI
br795		1	1	10	3	4	1	1	32	M4		VNI
ug2463		1	1	1	3	2	1	5	6	M10a		VNI
ug2471		1	1	10	3	2	1	1	31	M4b		VNI
H99		7	1	1	1	1	1	2	2	M1b		VNI
WM148		7	1	1	18	1	1	1	63	M1		VNI
WM626		2	14	14	8	11	11	27	97	M7		VNII
WM629		16	21	30	19	13	1	19	117			VNIV

Note: ^#^Meyer et al. [33]; ^∗^Litvintseva et al. 2006. ^1^Determined by URA5-RFLP analysis or M13 PCR-fingerprinting. ISHAM: international society for human and animal mycology; MLST: multilocus sequence typing; MLMT: multilocus microsatellite typing; ST: sequence type.

## Data Availability

The materials described in this work can be made available to interested researchers upon completion of the necessary agreements between institutions. Data generated for this study are included in the figures and additional materials.
